This article has been retracted.

# Personalized Teaching Strategy of University Ideology Course Based on Lagrange Neural Network and Big Data Technology

**DOI:** 10.1155/2022/1251839

**Published:** 2022-06-30

**Authors:** Jiqian Zuo, Fang Zhou, Yajuan Liang

**Affiliations:** ^1^College of Humanities and Marxism, Hebei Oriental University, Langfang 065001, China; ^2^College of Artificial Intelligence, Hebei Oriental University, Langfang 065001, China

## Abstract

Individualized instruction is a type of educational principle. On the one hand, it necessitates the creation of individualized teaching resources, courses, and methods. Students, on the other hand, require a high level of autonomy and the ability to make personalized plans based on their own cognitive characteristics and needs. The big data (BD) era opens up new possibilities for IE (ideological education) work in universities, but it also poses some challenges. IE development will be greatly aided by recognizing opportunities to meet challenges and optimizing and integrating PL (political lesson) resources. The LNN (Lagrange neural network) model has been established. The simulation results show that the LNN network can converge to the optimal solution quickly and effectively and then reconstruct sparse signals. Individualized college PL instruction using LNN and BD technology helps students communicate more effectively and improves the pertinence, immediacy, and positivity of IE.

## 1. Introduction

Massive data provide great value for people. Contemporary young students can be said to grow up together with the Internet [1, 2], so contemporary youth can be described as real participants and pioneers. The corresponding BD (big data) [3–5] era also has a profound impact on the education of universities. BD has brought profound changes to all fields. Faced with the great transformation power of BD, ideological teachers' way of thinking is bound to change, actively adapt to the requirements of the BD era, keep up with the times to the greatest extent, and make rational use of its advantages and characteristics to improve teaching effect.

Many large-capacity data sets are obtained from many large-scale data sets through intelligent statistical measures [6], and BD capacity exceeds traditional data storage capacity. Large capacity, fast processing speed, high total value, and diverse data types are all characteristics of BD [7]. The research on PL (political lesson) teaching mode innovation is also slightly involved, but the research results on BD's influence on college PL practice teaching are almost blank [8, 9]. As a result, when developing university PL personalization with a BD background, we must fully grasp BD's development opportunity, fully comprehend and grasp the theoretical hotspots and academic frontiers of college students' IE (ideological education) personalization by BD, and perfectly connect academic research results with actual teaching [10]. Universities' ideological staffs should focus on overcoming the dilemma of BD personalized teaching in the BD era, actively creating a variety of personalized teaching conditions.

The construction of teaching systems in research universities has given the teaching quality standard a new meaning and orientation. We should not only reflect the teaching quality standards of research universities in the index system of teaching evaluation but also reflect the teaching ideas of research education through the corresponding evaluation models, methods, and operating mechanisms when assessing classroom teaching quality. Finding new ways to do things has become a top priority. This paper examines the challenges faced by ideological network teaching resources and proposes optimization and integration methods to improve the teaching effect of ideological network teaching, based on the connotation and characteristics of BD.

## 2. Related Work

Literature [11] pointed out that the development of freshmen's online teaching should give priority to solving the problems of standardization and process, improving the platform of online education and teaching, and realizing the guarantee of infrastructure. Literature [12, 13] points out that with the popularization of online education and teaching in all parts of the country, many problems faced by online education and teaching are gradually exposed. Literature [14, 15] optimizes the current teaching mode by the BD method, provides teachers with information about students' learning behaviors and learning ways, and helps teachers understand the areas that students are good at and interested in. Literature [16] makes a preliminary study on personalized teaching and makes a superficial analysis of the influence of teachers' personalities and other factors on cultivating students from the perspective of establishing personalized consciousness and concept. Literature [17] studies the development process of personalized teaching from the perspective of teachers and puts forward that personalized teaching means that teachers fully integrate their own knowledge, experience, personality, and other factors with teaching activities to form a kind of teaching with unique style, stability, and personal characteristics of teachers. Literature [18] analyzes the personalized teaching mode by using the role theory and points out the premise guarantee and countermeasures of personalized teaching in combination with the opportunities and challenges faced by personalized teaching, so as to promote the teaching reform. Literature [19] holds that a personalized teaching classroom should be characterized by selectivity, daily life, and democracy, in which selectivity is the basic feature of personalized teaching, returning to students' life world is the essence of personalized teaching, and democracy is the premise and guarantee of personalized teaching.

In literature [20], a single-layer feedback neural network based on projection operation is proposed to solve the nonsmooth optimization problem with different objective functions. Literature [21, 22] puts forward a new type of neural network to solve general nonlinear programming problems. Literature [23] proposed a new type of neural network, LNN (Lagrange neural network), to solve nonlinear programming problems. Literature [24] studies the stability and convergence time of LNN in solving optimization problems. However, the objective functions of the optimization problems they solve are only smooth functions, so it is necessary to extend the application and research of this kind of neural network to nonsmooth optimization problems.

To summarize, online learning is attracting an increasing number of students due to its time and space flexibility as well as significant cost savings. With the rise of fragmented learning, customized and personalized online teaching based on BD has become the online teaching platform's development trend, providing a large number of potential users for BD in the development of online teaching, and the combination of BD and online teaching also has promising practices and research prospects.

## 3. Research Method

### 3.1. Personalized Instructional Design Based on BD

Personalized teaching is becoming a hot topic in China's educational circles as they try to reform the curriculum and change teaching methods. Because students differ in cognitive ability, cognitive level, and personality, educators should integrate students' personalities and teaching activities, put people first, begin teaching with students' needs, respect students' personalities, and use personalized teaching. Personalized teaching is a type of teaching idea that has three meanings: first, personalized teaching emphasizes the diversification of teaching, and teaching materials, teaching resources, teaching forms, and teaching methods should be rich and colorful; second, personalized teaching is learner-centered, values learners' subjectivity, respects students' individual differences, and meets students' diverse needs; and third, personalized teaching is learner-centered, attaches importance to learners' subjectivity, respects students' individual differences, and meets students' diverse needs.

The data of a learner's entire learning process can be recorded using BD technology. Knowledge points are assigned to every topic and data collected in tests, assignments, and exams. Encourage students to study more effectively and improve the quality of their learning. Various text and video resources can also be pushed to learners to help them internalize and absorb knowledge points. Students' learning motivation and interest are stimulated, and students' innovative, problem-solving, and practical abilities are developed. The implementation process is shown in Figure 1.

Through digital analysis to build a data model and use this resource to get students' psychological feelings during this period. For students who behave abnormally, find the source of the problem through data analysis and guide the wrong ideas in time.

At the same time, abundant IE resources and various forms of IE models provide students with a comprehensive platform for learning, which can satisfy students' personality styles and learning initiatives. Therefore, study in an online classroom or use WeChat to brainstorm and learn. In short, college PL teachers should comply with the development requirements of the BD era, further use BD to find favorable resources and information to master the IE initiative, and enrich and adjust teaching content with dynamic data. Before entering the course, connect and arrange the learning contents according to the key points and subkey points; at the same time, arrange your own learning time, which time period to learn what content, and when to conduct self-evaluation; and constantly revise your personal plan in combination with teachers' teaching.

On the one hand, independent assessment has no bearing on the teaching process. Only in an environment where teaching quality is highly valued and pursued can the evaluation result information be considered an integral part of school decision-making, and it is this information that the school administrators use. On the other hand, schools' value choice in using teaching evaluation results should be based on improving teachers' teaching ability, promoting teachers' development, then promoting students' development, fully mobilizing teachers' enthusiasm, and stimulating teachers' potential so that both teachers and students can benefit from teaching evaluation and so that teaching evaluation can be widely recognized and continuously promote the improvement of both teachers and students.

The penalty coefficient of LNN is variable, and the neural network can still converge to the optimal solution of the optimization problem without calculating the initial value of the penalty term in advance. A neural network model of differential inclusion is established to solve the optimization problem. The similarity calculation formula of the two nodes is

(1) $$\begin{array}{c} \text{sim}\left(U,U^{\prime }\right)=\sum_{i=1}^{n}w_{j}\cdot \text{sim}P{\left(U,U^{\prime }\right)}_{i}, \end{array}$$

where sim*P*_*i*_(*U*, *U*′) represents the similarity between node *U* and CN *U*′ and *w*_*j*_ represents the weight value of this attribute in the *i*-th attribute.

*MAXL* represents the length of the longest path in the tree and *P*(*a*_1_, *a*_2_) represents the distance between nodes. Therefore, the similarity calculation formula is:

(2) $$\begin{array}{c} {\text{sim}}_{cp}=\left(cp_{1},cp_{2}\right)=\frac{MAXL-\left|p\left(cp_{1},cp_{2}\right)\right|}{MAXL}. \end{array}$$

Teachers can assign different difficulty problems to students at different levels in class, which meets the individualized needs of students at each level, increases teaching efficiency, and truly realizes individualized teaching. Teachers can also gather students with problems in the same knowledge point based on the correct or incorrect situation of knowledge points and provide targeted explanations and training to help students improve and progress quickly. To help students master the content related to knowledge points, focus on synchronous or asynchronous explanations of common problems. Students can have individualized communication for personality issues. The explanation methods for students vary according to different knowledge points, which can promote the development of students' personalities and allow questions to be solved and answered at any time.

Personalized teaching based on BD can collect all of the students' data automatically; manage all types of learning materials digitally, such as students' homework, pictures, grades, and teachers' comments; track and record students' learning behaviors with BD technology; provide adaptive learning feedback; and provide students with personalized learning guidance. It is more convenient for students to think and reflect, objectively promote students' progress, and make students more active in self-evaluation by collecting and managing their entire process data.

### 3.2. Probe into the Personalized Teaching Path of University PL Based on LNN

Introducing the thinking mode of planning into college IE teaching based on BD is to break through the fixed thinking mode, with new eyes, new viewpoints, and new methods, from the establishment of the thinking mode of college IE planning to the implementation of the plan and the realization of the target requirements. Under the influence of BD, the way of IE in traditional mode has undergone great changes.

One is to accurately judge the resources of ideological network teaching, that is, the selected teaching resources can be authentic, effective, and reliable enough. The second is to find the best resources from massive IE resources, so as to ensure the best teaching effect. Of course, on the basis of the principle of scientific construction, should reach a certain degree of adaptability, specifically, the selected materials can adapt to students' physical and mental characteristics and knowledge structure characteristics. This work should also pay attention to two points: one is to choose the teaching resources that fit the students' actual network, and the other is to seriously explore the students' concerns and interests and find out the places where students have insufficient knowledge to enhance the pertinence of the teaching process.

The goal of this paper is to design a neural network so that its equilibrium point can meet the optimal conditions. In order to explain the neural network model, firstly, a Lagrangian-like function is defined as follows:

(3) $$\begin{array}{c} L\left(x,\lambda \right)=f\left(x\right)+\lambda H\left(x\right). \end{array}$$

in which Lagrange multiplier *λ* > 0.

(4) $$\begin{array}{c} H\left(x\right)=\left\{\begin{array}{cc} 0, & x\in S,\\ \sum_{j\in I^{+}\left(x\right)}h_{j}\left(x\right), & x\notin S. \end{array}\right) \end{array}$$

Find the *L*_1_(*x*, *λ*)-square *x*-guide number of the Lagrange function:

(5) $$\begin{array}{c} \nabla_{x}L\left(x,\lambda \right)=\partial f\left(x\right)+\lambda^{T}\nabla h\left(x\right). \end{array}$$

According to the gradient descent, the following neural network can be constructed:

(6) $$\begin{array}{c} \left(\begin{array}{c} \frac{\text{d}x}{\text{d}t}=-\nabla_{x}E=-\nabla_{x}f\left(x\right)-\lambda A-\mu A^{T}\left(Ax-b\right)\\ \frac{\text{d}\lambda }{\text{d}t}=\nabla_{\lambda }E=Ax-b \end{array}\right\}. \end{array}$$

Because the operator ‖·‖_0_ is not differentiable, the function *f*(*x*_*i*_) ≈ *x*_*i*_^2^/*x*_*i*_^2^+*σ* is considered to approximate ‖*x*‖_0_. The smaller *σ* is, the more accurate the approximation effect is, that is:

(7) $$\begin{array}{c} {\left\|x\right\|}_{0}\approx f\left(x\right)=\sum_{i=1}^{n}f\left(x_{i}\right)=\sum_{i=1}^{n}\frac{x_{i}^{2}}{x_{i}^{2}+\sigma }. \end{array}$$

Differentiated assessment is possible thanks to the teaching cloud platform's ability to personalize curriculum assessment strategies for different classes. Most students who major in art or sports, for example, are outgoing and good communicators, but they dislike reading. College PL teachers can focus on content material learning and knowledge consolidation exercises and strive to help students lay a strong theoretical foundation and develop a practical learning attitude, depending on their characteristics. Create more personalized practice plans and improve the methods and forms of practice. Personalized practice schemes can effectively stimulate students' interest in learning, arouse participation in practical activities, and improve their overall creative ability in the relatively relaxed, happy, and free practice process.

Evaluate and judge the similarity between the given user portrait model and the user portrait model in the user portrait database. The user's current learning user portrait is called the main learning user portrait. The user portrait similarity calculation obtains the user portrait similarity by constructing a decision tree and performing node operation. Taking the user attribute elements as an example, the user portrait model tree is constructed, as shown in Figure 2.

Teachers' personalized teaching system is used to watch the completion and accuracy of students' preview self-test questions. Because each test question has different knowledge points, the students' mastery degree is analyzed to understand the overall preview of students. According to the real-time updated ranking of students' preview scores, this paper analyzes the changes in students' grades and the wrong questions of each student, so as to teach students in accordance with their aptitude in the process of teaching.

Cloud engine in BD infrastructure module realizes the management of distributed Hadoop nodes through task scheduling function. Considering that other modules in the system, such as database management module of user portrait, also need to manage the database by task scheduling, asynchronous task transfer is adopted, which also ensures the rapid development and debugging of submodules as shown in Figure 3.

The script is developed in python, which mainly includes two parts, task and task fragment. The task is initialized in the management server by reading the policy file, and the task script and shell script are packaged according to the corresponding configuration in the policy file. After the packaging is completed, it is sent to the proxy service module of the Hadoop node through socket. The proxy service module decompresses the task and shell script, executes the task fragment script, calls the corresponding shell script, completes the task scheduling, and returns the execution result to the cloud engine.

Individualized teaching creates a democratic and harmonious atmosphere for teachers and students and allows students to have their own thoughts and answers, thus fully expressing their individuality. Personalized teaching is personalized in curriculum, teacher's teaching, and students' learning. Mind mapping also reflects personalization. Deal with the problem according to the way you handle the information, which obviously has a strong personal color. When thinking or solving problems and combine multidimensional information into a dynamic structure diagram, what is completed is a personalized mind map.

## 4. Results Analysis and Discussion

Under BD background, IE personalized teaching needs the comprehensive strength of teachers and technical teams. Specifically, the construction of a personalized teaching team can improve BD development literacy through the optimization and potential stimulation of the internal staff of the teaching team and strengthen the screening and optimization of massive teaching data. It can focus on future development education and fully absorb data professionals from all aspects to strengthen personalized teaching. This innovative personalized teaching method can gradually transform the traditional IE work from the extensive passive response mode to the active intervention and active guidance mode and create a new personalized teaching mode of college IE.

Using MATLAB to generate sparse signal *x* of order *k*, without losing generality, the positions of these *k* nonzero elements are randomly generated and meet the uniform distribution of [1, *n*], and the sizes of the corresponding nonzero elements are randomly generated and meet the uniform distribution among [1, 100]. The generation of random signals is shown in Figure 4.

Students' intuitive and comprehensive qualitative evaluation of teachers and courses is referred to as aspect evaluation. The individual evaluation reflects the quantitative requirements for teaching based on subject characteristics or course nature. Teachers' personal styles and preferences, as well as the school's current reform focus, are reflected in the selective evaluation. Subjective evaluation captures characteristics of teaching quality that aren't captured by standardized indicators. Teachers can also use a specific knowledge point or piece of content as a theme for each group to investigate and promote. Teachers can allow students to create their own personalized mind map during the evaluation stage, which includes not only the relationships between knowledge points but also their own learning methods and cognitive strategies. Students can use this map to learn about their learning situation and provide timely feedback, making it easier for them to identify and correct their own flaws, humanize the evaluation, and make the cognitive and thinking processes operable.

Virtual practice teaching alleviates the difficulties of traditional practice teaching, such as students' lack of subjectivity, limited teaching time and space, shortage of teaching resources, and so on; highlights students' dominant position; expands the field of teaching virtual space; and enriches teaching resources. In the course system construction of personalized teaching, the setting of emotion and belief courses cannot be ignored. A complete personalized teaching course system should be the integration of three courses. Therefore, on the basis of the main courses, emotion and belief courses should be properly arranged, and at the same time, emotion courses should be refined into the specific teaching of the first two courses. Teachers can link the first two courses with the third related part in teaching; for example, they are often combined with corresponding emotions in the teaching of psychology, and the beliefs and thoughts of historical figures are linked with them in the teaching of anthropology so that the three courses are harmonious and unified.

In order to test the relationship between the observation times *m* and the correct reconstruction probability under different sparsity, take different sparsity *k*=[10,15,20,25] and perform 1,000 random experiments on each group of (*k*, *m*, *n*).

It can be seen from Figure 5 that for different sparsity *k*, when the number of observation points *m* is greater than or equal to 110, the probability that LNN method can correctly recover sparse signals is extremely high.

The integration of BD and teaching is conducive to strengthening the supervision and management of college students' ideological fields. Through the digital analysis of students' ideological status, to control the operating mechanism of ideological education in colleges and universities, introduce new thinking ways and teaching methods, integrate the working resources of college IE, give full play to the advantages of digital technology, and cultivate the ability of college ideological educators to use data. Enhance the scientificity and modernity of college IE.

BD should be introduced into practice teaching, and more space for students to choose independently should be reserved in the PL teaching practice theme design. This can effectively stimulate students' initiative of independent innovation in the process of stimulating students' personal development potential. In the BD development environment, it can provide differentiated teaching ideas for college PL teaching and realize individualized education development. In personalized education, pay attention to actively listening to students' opinions and suggestions, praising students' personal strengths, which can safeguard students' personal dignity and interest.

As can be seen from Figure 6, for *m*=[10,15,20,25] with different observation points, when the sparsity *k* is less than or equal to 20, the LNN method has a very high probability of correctly recovering sparse signals.

Provide training, expert guidance, and technical support for teachers to help them improve their teaching level. Establish a website for the purpose of “serving teachers' teaching” to provide teachers with places for learning and communication. Organize a series of discussion lectures and classroom observations to help young teachers learn from other teachers' advanced teaching experiences and form their own teaching style and characteristics. Hire experienced old teachers as teaching consultants, listen to young teachers' classes regularly, and give guidance. Carry out a series of educational technology training to improve teachers' ability to master modern technologies such as multimedia.

The visualization of a mind map can help students understand the solutions and methods adopted by teachers and classmates when solving the same problem. At the same time, continuous reflection and regulation can promote the formation and transfer of their own cognitive strategies and cultivate their metacognitive ability. The explicit way of mind map opens tacit knowledge, realizes information exchange, connects more information to expand the breadth and depth of thinking, inadvertently exercises thinking, and lays the foundation for the emergence of new inspiration and the stimulation of creativity, thus promoting the innovation and perfection of knowledge.

Use MATLAB software programming to simulate the behavior of the neural network.  Figure 7 shows the trajectory diagram of *x*_1_, *x*_2_.  Figure 8 shows the trajectories in these four points *x*_1_. Therefore, this is consistent with the minimum point set in problem analysis.

Learning objectives have a specific order, and they do not exist in parallel. Similarly, knowledge points follow a logical order: before learning a specific knowledge point, you must first learn its lower knowledge points, which serves as a necessary prelude to learning the upper knowledge points and improving the upper knowledge points. Students will be pushed to master the basic knowledge points, then the writing knowledge points of chemical equations, and finally the knowledge points related to the simple calculation of chemical equations. Students will master knowledge content ranging from easy to difficult, and personalized learning will be realized. There are two types of personalized teaching resources: static and dynamic. Words, pictures, animations, courseware, and material conditions are examples of static resources, whereas dynamic resources refer to dynamic information and active human resources. The construction of static resources is currently mostly in the stage of low-level repeated construction in the resource creation process, and the lack of individuality cannot meet the needs of students. Furthermore, it frequently overlooks the discovery of dynamic resources hidden in teaching activities, such as creativity and intellectual resources. However, mind maps can assist in the resolution of these issues.

It can be seen from Figure 9 that the initial point (*x*_1_=1, *x*_2_=0.5) inside the feasible region finally converges to the minimum point. It can be seen from Figure 10 that the initial point (*x*_1_=0, *x*_2_=5) outside the feasible region enters the feasible region after a period of operation and finally converges to the minimum point (*x*_1_=0, *x*_2_=2).

In order to facilitate code maintenance and subsequent expansion of functions, Python and Shell scripts that can explain execution are selected. When running on the system line, the code can be modified. The task dispatching room executes in sequence through queues, and the cloud engine executes corresponding tasks according to the priority of the queues. So the elements that make up the user portrait must be able to be automatically identified by the computer, or the user can provide explicit information about the elements of the user portrait. When building a user portrait model, the finer the entity elements that make up the model, the more accurate the description of the model is. However, in the actual application process, many and fine user portrait elements will be dull. Therefore, the scope and accuracy of the user portrait model must meet the actual needs.

The platform will continuously collect user information and apply it to the current user portrait and constantly improve the user's portrait features through the current user portrait's use of data, so as to realize the continuous enrichment and perfection of data and portrait and ensure that the model has good adaptability. According to the difference of data dimensions, starting from multidimensions, the data is finally aggregated into a cluster set with the least differentiation in a certain dimension. There are often great differences between different clusters, so cluster analysis has become a commonly used data processing method in the field of machine learning.

## 5. Conclusion

Students have more autonomy with personalized instruction. They will not get the corresponding effect if they are too free, so educators, particularly front-line teachers, must grasp and control it properly. Furthermore, no idea or tool can be flawless. We can make them work by constantly exploring and tapping their useful value. When incorporating the LNN development concept into university PL personalized teaching, it is important to keep in mind that students' personalized development differs. Encourage students to actively change their learning styles, pique their curiosity about learning, and develop their practical skills and creative spirit. Establish and improve the incentive and restraint mechanisms in the classroom, as well as stimulate teachers' awareness of the need to continually improve teaching and their level of expertise. The outcome of classroom evaluation is useful for postappointment teaching, professional and technical postappointment, and various awards.

## Figures and Tables

**Figure 1:** Implementation flow chart.

**Figure 2:** Schematic diagram of user attribute tree.

**Figure 3:** Working mechanism of task submodule.

**Figure 4:** Discrete sparse signal.

**Figure 5:** The relationship between the measured number *m* and the probability of successful recovery.

**Figure 6:** Relationship between sparsity *k* and probability of successful recovery.

**Figure 7:** *x*_1_, *x*_2_ trajectory.

**Figure 8:** Trajectory of any four initial points *x*_1_.

**Figure 9:** Trajectory of state vector *x*(*t*) with an initial point in the feasible region.

**Figure 10:** Trajectory of state vector *x*(*t*) of an initial point outside the feasible region.

## Data Availability

The data used to support the findings of this study are available from the corresponding author upon request.

## References

[1] Wang W., Chen D. (2017). Analysis on the innovation path of ideological and political theory courses in colleges and universities in the big data era. *Ideological Education Research*.

[2] Lu Q., Li C. (2021). Synergy: the coupling development of big data and ideological and political theory courses in colleges and universities. *School Party Building and Ideological Education*.

[3] Jin X.-B., Gong W.-T., Kong J.-L., Bai Y.-T., Su T.-L. (2022). PFVAE: a planar flow-based variational auto-encoder prediction model for time series data. *Mathematics*.

[4] Cai W., Song Y., Wei Z. (2021). Multimodal Data Guided Spatial Feature Fusion and Grouping Strategy for E-Commerce Commodity Demand Forecasting. *Mobile Information Systems*.

[5] Jin X.-B., Gong W.-T., Kong J.-L., Bai Y.-T., Su T.-L. (2022). A variational bayesian deep network with data self-screening layer for massive time-series data forecasting. *Entropy*.

[6] You L., Jiang H., Hu J. (2021). GPU-accelerated Faster Mean Shift with Euclidean Distance Metrics. https://arxiv.org/abs/2112.13891.

[7] Wu Y. (2020). Research on the application of big data technology in ideological and political education in the information age——comment on “big data and ideological and political theory courses in colleges and universities”. *Chinese Science and Technology Paper*.

[8] Yu W. (2021). Research on the combination of big data and ideological and political education for college students——comment on “theory and practice of ideological and political education in higher vocational courses in the new era”. *Science and Technology Management Research*.

[9] Zhang N. (2021). Exploration of the informatization of ideological and political education in colleges and universities in the era of big data——comment on “theory and practice of flipped classroom in ideological and political courses in colleges and universities in the Internet era”. *Science and Technology Management Research*.

[10] Liu R. (2021). Analysis on the stratified intervention of mental health education in colleges and universities. *ASP Transactions on Psychology and Education*.

[11] Zhang L. (2018). Innovating personalized ideological and political education in colleges and universities in the era of big data. *China Higher Education*.

[12] Wang W., Liu X. (2020). Accurate academic guidance for colleges and universities in the era of big data: paths, conditions and reflections. *Educational Exploration*.

[13] Wang X. (2019). Research on teaching reform based on educational big data. *Educational Theory and Practice*.

[14] Zhou H., Yi L. (2017). The reform of teacher education in the era of big data. *Educational Research and Experiment*.

[15] Wang J. (2017). Ruiyi Cloud Teaching——using the cloud platform for personalized teaching. *People’s Education*.

[16] Song Y., Guo J. (2017). Neuro-adaptive fault-tolerant tracking control of Lagrange systems pursuing targets with unknown trajectory. *IEEE Transactions on Industrial Electronics*.

[17] Qiang X., Zeng Z. (2017). Scale-limited Lagrange stability and finite-time synchronization for memristive recurrent neural networks on time scales. *IEEE Transactions on Cybernetics*.

[18] Sun Y., Chen L., Ma G., Li C. (2017). Adaptive neural network tracking control for multiple uncertain Euler-Lagrange systems with communication delays. *Journal of the Franklin Institute*.

[19] Huang Y., Yuan X., Yang X., Long H., Xiao J. (2020). Multiple Lagrange stability and Lyapunov asymptotical stability of delayed fractional-order Cohen–Grossberg neural networks. *Chinese Physics B*.

[20] Sheng Y., Lewis F. L., Zeng Z., Huang T. (2019). Lagrange stability and finite-time stabilization of fuzzy memristive neural networks with hybrid time-varying delays. *IEEE Transactions on Cybernetics*.

[21] Jia C., Wang D., Yin J., Chen X., Zhang L. (2018). Joint multiple sources localization using TOA measurements based on Lagrange programming neural network. *IEEE Access*.

[22] Li L., Li C. (2019). Discrete analogue for a class of impulsive cohen-grossberg neural networks with asynchronous time-varying delays. *Neural Processing Letters*.

[23] Bober D. B., Lagrange T., Kumar M., Rupert T. J. (2019). Pronounced grain boundary network evolution in nanocrystalline Cu subjected to large cyclic strains. *Journal of Materials Research*.

[24] Tu Z., Wang D., Yang X., Cao J (2020). Lagrange stability of memristive quaternion-valued neural networks with neutral items - ScienceDirect. *Neurocomputing*.

